# Silencing SUMO2 promotes protection against degradation and apoptosis of nucleus pulposus cells through p53 signaling pathway in intervertebral disc degeneration

**DOI:** 10.1042/BSR20171523

**Published:** 2018-06-29

**Authors:** Liu-Zhong Jin, Ji-Shou Lu, Jian-Wen Gao

**Affiliations:** Department of Spine Surgery, Jining No. 1 People’s Hospital, Jining 272000, P.R. China

**Keywords:** Intervertebral disc degeneration, Nucleus pulposus cells, p53 signaling pathway, Proliferation, SUMO2 gene silencing

## Abstract

Objective: Intervertebral disc degeneration (IDD), as a common cause of back pain, is related to the promotion of cellular senescence and reduction in proliferation. Based on recent studies, small ubiquitin-related modifier (SUMO) proteins have been implicated in various biological functions. Therefore, in the present study, we investigated the effects of SUMO2 on proliferation and senescence of nucleus pulposus cells (NPCs) via mediation of p53 signaling pathway in rat models of IDD.

Methods: After the establishment of rat models of IDD for the measurement of positive expression of SUMO2/3 protein, the mRNA and protein levels of SUMO2, molecular phenotype [matrix metalloproteinase-2 (MMP-2) and hypoxia-inducible factor-1α (HIF-1α)] and p53 signaling pathway-related genes [p21, murine double minute-2 (MDM2), growth arrest and DNA-damage-inducible protein 45 α (GADD45α), cyclin-dependent kinase 2/4 (CDK2/4), and CyclinB1] were determined, followed by the detection of cell proliferation, cell cycle, apoptosis, and cell senescence.

Results: The rat models of IDD were successfully constructed. The results obtained showed that there was a higher positive expression of SUMO2/3 protein in IDD rats. Moreover, the silencing of the SUMO2 gene decreases the levels of SUMO2, p53, p21, MDM2, GADD45α, MMP-2, and HIF-1α expressions and p53 phosphorylation level while it increases the levels of CDK2/4 and CyclinB1 expressions. In addition, SUMO2 gene silencing enhances proliferation and suppresses apoptosis and cell senescence of NPCs.

Conclusion: In conclusion, SUMO2 gene silencing promotes proliferation, and inhibits the apoptosis and senescence of NPCs in rats with IDD through the down-regulation of the p53 signaling pathway. Thus, SUMO2 is a potential target in the treatment of IDD.

## Introduction

Intervertebral discs are pads of fibrocartilage, located between the vertebral body of the spine with degenerative changes, which are a major cause for back pain associated with aging [1]. Intervertebral disc degeneration (IDD) is regarded as a complex process accompanied by age-related change and tissue damage caused by stress, which is closely related to the promotion of cellular senescence, inflammatory response and catabolic metabolism, and reduced proliferation [2]. IDD, which is known to be asymptomatic in many cases, is closely associated with disc herniation, spinal stenosis, and radicular pain resulting from imbalance between catabolic and anabolic responses [3,4]. Although numerous therapeutic methods have been introduced for the treatment of IDD, including gene therapy, cell therapy and biological therapy, [5–7] the underlying molecular mechanism of IDD is yet to be fully identified [2].

The SUMO2 protein family is a family of 17 kDa in mammals and one member in the yeast *Saccharomyces cerevisiae*, which has a functional value in the regulation of a large number of target molecules [8]. There are three members in the SUMO family including SUMO1, SUMO2 and SUMO3, which are conjugated as post-translational modifications to target proteins [9]. Meanwhile, the conjugation of SUMO into specific proteins is a new modulation for post-translational process in almost all cellular physiology [10]. Sumoylation pathways were expressed in IVD cells and localized predominantly in nuclei. Emerging evidence showed that in NP cells hypoxia transiently increased the expression of SUMO-1 and SUMO-2/3 [10]. The role of SUMO molecules in IDD remains to be elucidated. Furthermore, a previous study has revealed that p53 signaling pathway exerts great effects on the senescence of cartilage end plates (CEP) cells involved in IDD [11]. It has also been reported that p53 could be regulated by SUMO [12]. p53, a well-known tumor suppressor in humans and other mammals, mainly functions as a transcription factor, which can positively or negatively regulate a number of responsive genes [13]. The activation of p53 that has been modified by SUMO is closely related to the onset of cellular senescence [14]. The results from the present study revealed that SUMO2 gene silencing mediated the p53 signaling pathway to ameliorate or postpone IDD by promoting the proliferation of nucleus pulposus cells.

## Materials and methods

### Ethical statement

The animal experimental processes were approved by the Ethnic Committee of Jining No. 1 People’s Hospital and conducted in strict accordance to the standard of the Guide for the Care and Use of Laboratory Animals published by the Ministry of Science and Technology of the People’s Republic of China in 2006.

### Animal grouping and modeling

A total of 40 healthy male Sprague Dawley (SD) rats (weight 200–250 g) were purchased from experimental animal center of the fourth military medical university. Following a one-week adaptive feeding, the rats were classified into the IDD (*n*=30) and sham (*n*=10) groups. After the rat model had been established using acupuncture therapy of anulus fibrosus (AF), the rats in the IDD group were intraperitoneally anesthetized using 3% pentobarbital sodium (Hubei Hong Yunlong Biotechnology Co., Ltd., Wuhan, China) at a dose of 30 mg/kg. After the rats were shaved and fixed, their left side was disinfected and then covered with aseptic towel. A 2-cm incision was made on the posterior part of the right abdomen along the back muscles and musculus obliquus externus abdominis. According to the localization of iliac crest, the L3-4, L4-5, and L5-6 intervertebral space was exposed from the extraperitoneal approach to the right side of the vertebral body. A 16 G puncture needle was used to pierce into L4-5 intervertebral space at an angle of 45° on the spine sagittal plane and anterolateral parallel plate of intervertebral disc AF, and a full-layer acupuncture was conducted at 2.3 mm for 10 s. After withdrawal of needles, the wound was sutured. As for the sham group, the suturing was done immediately after the incision. Rats in the two groups were injected with penicillin sodium at 200,000 U/kg (North China Pharmaceutical Co., Ltd., Shijiazhuang, China) once a day, within the abdomen to prevent infection. The rats in each group were placed in an environment with a temperature of 23–25°C and followed a normal consistent feeding habit for 6 weeks. The morphological and pathological changes of the intervertebral discs were observed in the IDD group and the sham group respectively to check for a successful model establishment. Out of the 40 rats, ten rats were killed during the modeling process (one in the sham group and nine in the IDD group).

### Pathology of intervertebral disc

Two rats were randomly selected from the IDD group and sham group and were executed through an intraperitoneal injection of excessive anesthesia. The intervertebral disc specimens were extracted from the interface between the vertebral body and the upper and lower cartilage end plates. The specimens were dehydrated by gradient ethanol and cleared by xylene. Subsequently, the paraffin-embedded specimens were sliced into 4-μm serial sections. Both the sham and IDD groups had two pieces of specimens. The experiment was repeated three times. Then, the sections were stained with hematoxylin (Beijing Solarbio Science & Technology Co., Ltd., Beijing, China) solution for 10 min and washed with water twice, 1 min for each session. Then, they were differentiated with 1% hydrochloric acid alcohol for 30 s and washed with water twice. The sections turned back to blue using weak ammonia water for 15 s, and washed with water for 3 min. After staining with 0.5% eosin alcohol (Beijing Solarbio Science & Technology Co., Ltd., Beijing, China) for 3 min, the sections were washed with water for 2 min and subsequently, dehydrated, cleared, and sealed. The sections of the model and sham groups were observed at the same location using an optical microscope (EcliPse.E2OO, Nikon, Japan). The changes of collagen fibers in NPCs and nucleus pulposus were observed by JEM-1230 transmission electron microscope (Japan Electronics Corporation, Japan).

### Immunohistochemistry

Two rats were randomly selected from both the model and sham groups. They were treated with heart perfusion of paraformaldehyde after anesthesia. Subsequently, the intervertebral disc on the modeling section was immersed in paraformaldehyde for 24 h, followed by conventional sections, with two sections in the model and sham groups respectively. The experiment was performed in triplicate. After antigen retrieval was conducted using a microwave oven, the sections were treated with 3% hydrogen peroxide to block endogenous peroxidase. The sections were added with SUMO2/3 primary antibody (ab109005, 1:100, rabbit antibody, Abcam Inc., Cambridge, U.K.) and were left for incubation overnight in the refrigerator at 4°C. Next, polymerase adjuvant was added to the sections before incubation for 20 min at room temperature, followed by the addition of goat anti-rabbit secondary antibody (ab6721, 1: 2000, goat antibody, Abcam Inc., Cambridge, U.K.) for incubation at room temperature for 30 min. The sections were stained with diaminobenzidine (DAB, ab64238, Abcam Inc., Cambridge, U.K.), and the nucleus was counterstained with hematoxylin. Afterward, the sections were dehydrated, cleared, and sealed and the number of SUMO2/3 protein positive cells was counted using a CX31-LV320 microscope (Olympus Optical Co., Ltd, Tokyo, Japan) at the same position, and the cells that appeared to be like brown particles were identified as the positive cells.

### Isolation, purification, and identification of NPCs

After the rats had been fed for 6 weeks, the remaining rats were killed through an intraperitoneal injection of excessive anesthesia. After isolation, the gelatinous nucleus pulposus was obtained and rinsed three times with D-HanK’s solution. The tissues were sliced into 1 mm × 1 mm × 1 mm pieces, which were transferred into centrifuge tube for digestion with type II collagenase for 2 h, followed by centrifugation at 1000 rev/min and removal of the supernatant. Next, the cells were digested with hyaluronidase (10 U/ml) in water bath for 2 h followed by centrifugation at 1000 rev/min and washing three times with Dulbecco’s Modified Eagle Medium (DMEM)/F12 (Gibco Company, Grand Island, NY, U.S.A.). Then, they were inoculated in DEME/F12 medium containing streptomycin (100 U/ml) and 10% fetal bovine serum (FBS) (Four Seasons Green Biology Institute, Hangzhou, China), followed by conventional culture with 5% CO_2_ at 37°C. Next, the cells were treated with digestion and passage once within 2–3 days. The morphological changes of NPCs in primary and passaged IDD rats were observed under the CKX41-A32PH phase contrast inverted microscope (Olympus Optical Co., Ltd., Tokyo, Japan).

The second generation cells were taken for cell climbing and fixed in 4% paraformaldehyde at room temperature for 30 min. Subsequently, the sections were rinsed three times with phosphate buffered solution (PBS), 5 min each time, followed by incubation with 3% H_2_O_2_ at room temperature for 15 min. After being washed with PBS for three times, 5 min each time, the sections were added with citrate buffer (0.01 mol/l) for repairing at 95°C for 15 min and rinsed with PBS three times, 5 min each time, after the sections were cooled. Subsequently, the sections were blocked with 5% goat serum sealing fluid at 37°C for 30 min followed by the addition of rabbit anti-rat type II collagen (1:100, Bios Biotechnology Co., Ltd., Beijing, China) before incubation overnight at 4°C. After washing with the PBS three times, 5 min each time, the sections were added with the biotin-labeled secondary antibody, followed by incubation at room temperature for 30 min. Afterward, the sections were washed with PBS three times, 5 min each time, and were stained with DAB for 5 min, counterstained with hematoxylin, sealed with neutral resin, and observed under an optical microscope.

### Construction of lentivirus vector

Three pairs of shRNA primers used in the interference of the SUMO2 gene were designed according to the instructions of PLL3.7 cloning vector and were annealed to double-stranded DNA for later use. The SUMO2 shRNA and PLL3.7 vectors were digested and linked with the same restriction endonucleases and the resultant plasmids were named PLL-SUMO2-shRNA1, PLL-SUMO2-shRNA2, and PLL-SUMO2-shRNA3 respectively. For the transformation of the plasmids into *Escherichia coli* DH-5α competent cells, a One-step transformation was performed, followed by the extraction of plasmids. The NPCs in the logarithmic growth phase in the sham group were inoculated into a 12-well plate with 1.2 × 10^6^ cells per well, which were randomly distributed into the PBS, PLL-SUMO2-shRNA1, PLL-SUMO2-shRNA2, and PLL-SUMO2-shRNA3 groups in triplicate. The interfering plasmid (or PBS) (0.5 μg) and packaging vector (PG a g/Pol, PVSV-G and PRev) (1.5 μg) were mixed with the lentiviral packaging system. The mixture was cotransfected into the NPCs in corresponding groups. Following transfection for 48 h, the NPCs in the four groups were observed by a fluorescence microscope to determine the expression of green fluorescent protein. After transfection for 72 h, the samples were centrifuged and filtered with the virus supernatant and were stored for further use. The primer sequences for SUMO2-shRNA are displayed in Table 1.

**Table 1:** SUMO2-shRNA primer sequences

Gene	Primer Sequences (5′-3′)
shRNA1	Sense strand: 5′-CCGGCCTATTGTGAACGACAGGGATCTCGAGATCCCTGTCGTTCACAATAGGTTTTTG-3′
	Antisense strand: 5′-AATTCAAAAACCTATTGTGAACGACAGGGATCTCGAGATCCCTGTCGTTCACAATAGG-3′
shRNA2	Sense strand: 5′-CCGGGAGGCAGATCAGATTCCGATTCTCGAGAATCGGAATCTGATCTGCCTCTTTTTG-3′
	Antisense strand: 5′-AATTCAAA AAGAGGCAGATCAGATTCCGATTCTCGAGAATCGG AATCTGATCTGCCTC-3′
shRNA3	Sense strand: 5’-CCGGGCACAGTTGGAAATGGAGGATCTCGAGATCCTCCATTTCCAACTGTGCTTTTTG-3′
	Antisense strand: 5′-AATTCAAAAAGCACAGTTGGAAATGGAGGATCTCGAGATCCTCCATTTCCAACTGTGC-3′

Abbreviation: SUMO2, small ubiquitin-related modifier 2.

### Cell grouping and transfection

The experiment was assigned into the sham (the 35th generation NPCs from rats in the sham group), model (the 35th generation NPCs from rats in the IDD group transfected without lentivirus), negative control (NC) (the 35th generation NPCs from rats in the IDD group transfected empty lentivirus), shRNA1 (the 35th generation NPCs from rats in the IDD group transfected with PLL-SUMO2-shRNA1 lentivirus), shRNA2 (the 35th generation NPCs in the IDD group transfected with PLL-SUMO2-shRNA12 lentivirus), and shRNA3 (the 35th generation NPCs from the rats in the IDD group transfected with PLL-SUMO2-shRNA3 lentivirus) groups. A total of 20 pmol Lipofectamine^TM^ 2000 (Invitrogen Inc., Carlsbad, CA, U.S.A.) (the sham and IDD group), empty lentivirus, PLL-SUMO2-shRNA1 lentivirus, PLL-SUMO2-shRNA2 lentivirus, and PLL-SUMO2-shRNA3 lentivirus were diluted with 50 μl of OPti-MEM and incubated at room temperature for 5 min. After dilution, the fluid was mixed with Lipofectamine^TM^ 2000 and placed at room temperature for 20 min. The cells were seeded in a 24-well plate with 4 × 10^4^ cells per well, with four wells in each group. When the cell proliferation reached 50%, 100 μl of the corresponding mixture was added and the solution went through incubation for 8 h. Subsequently, DMEM/F12 medium (containing 10% FBS) was replaced and incubated at 37°C in a cell incubator with saturated humidity with 5% CO_2_ for 48 h.

### Reverse transcription quantitative polymerase chain reaction (RT-qPCR)

SYBR Green method was adopted to determine the mRNA expression of SUMO2, phenotypic molecules [matrix metalloproteinase-2 (MMP-2) and hypoxia-inducible factor-1α (HIF-1α)] and genes related to p53 [p21, murine double minute-2 (MDM2), growth arrest, and DNA-damage-inducible protein 45α (GADD45α), cyclin-dependent kinase 2/4 (CDK2/4), and CyclinB1]. After the total RNA was extracted from cells in each group using a Trizol kit (RP2401, Beijingbai Teke Biotechnology Co., Ltd., Shanghai, China), colorimetric method was performed to determine the absorbance of *A*_260_/*A*_280_ ratio and the total RNA concentration. The total RNA was reversely transcripted to cDNA based on the instructions of reagent kit from Takara (Tokyo, Japan). The reaction conditions were as follows: at 37°C for 1 h, at 95°C for 5 min, and at 4°C perpetually. Subsequently, RT-qPCR was conducted (PH-K-100, Wuxi Bodhi Biomedical Technology Co., Ltd., Jiangsu, China), and the reaction system were as follows: SYBR GREFN Mix (5 μl), forward primer (1 μl), reverse primer (1 μl), cDNA (6 μl), RNase Free dH_2_O (10 μl). PCR amplification conditions were as follows: 30 cycles of at 95°C for 30 s, at 95°C for 5 s, at 58°C for 5 s, and at 65–95°C for 5 s. Glyceraldehyde phosphate dehydrogenase (GAPDH) was selected as the internal reference. The primer sequences are as shown in Table 2. The 2 (−Δ*C*_t_) method was used for the evaluation of mRNA expression of SUMO2 and to screen the lentiviral vectors with the best silencing effect which were named as the shRNA group. The relevant molecular mRNA expression test was carried out in the shRNA group, and the experiment was repeated three times. The following experiment was also conducted in this group.

**Table 2:** Primer sequences for RT-qPCR

Gene	Primer sequences (5′-3′)
p53	Forward: GACGCTGCCCCCACCATGAG
	Reverse: ACCACCACGCTGTGCCGAAA
p21	Forward: GGCAAGAGTGCCTTGACGAT
	Reverse: AAGAAAGCCCTCCCCAGTTC
SUMO2	Forward: GGCAACCAATCAACGAAACAG
	Reverse: TGCTGGAACACATCAATCGTATC
GADD45α	Forward: TGCTCAGCAAGGCTCGGAGT
	Reverse: GTTGCTGACCCGCAGGATGT
CDK2	Forward: CATTCCTCTTCCCCTCATCA
	Reverse: GTACGGACAGGGACTCCAAA
CDK4	Forward: TTTGATCTCATTGGATTGCC
	Reverse: AGGTCAGCATTTCCAGCAG
CyclinB1	Forward: CGACAACTGGAGGAAGAGCA
	Reverse: ATGGTCTCCTGAAGCAGCCT
MDM2	Forward: CGGCCTAAAAATGGTTGCAT
	Reverse: TTTGCACACGTGAAACATGACA
MMP-2	Forward: ACCGTCGCCATCATCAA
	Reverse: CCTTCAGCACAAAGAGGTTGC
HIF-1α	Forward: ACAGTGGTACTCACAGTCGG
	Reverse: CCCTGCAGTAGGTTTCTGCT
GAPDH	Forward: CTGGTGCTGAGTATGTCGTGGA
	Reverse: AGTTGGTGGTGCAGGATGCATT

Abbreviations: CDK, cyclin-dependent kinases; GADD45α, growth arrest and DNA damage inducible 45α; GAPDH, glyceraldehyde-3-phosphate dehydrogenases; HIF-1α, hypoxia-inducible factor-1α; MDM, mouse double minute; MMP, matrix metalloproteinase; RT-qPCR, reverse transcription quantitative polymerase chain reaction; SUMO2, small ubiquitin-related modifier 2.

### Western blotting

Total cell proteins were extracted from the sham, model, NC and shRNA groups, and precooled with PBS. The cells were washed three times, 1 min each time. A total of 400 μl cell lysate (including benzyl sulfonyl fluoride) were added in each bottle. After the blotting was performed, the cells were split for 30 min, during which cells were oscillated for 30 s every 5 min. Subsequently, cells were centrifuged at 12000 rev/min at 20°C for 20 min, and supernatant was collected with a new centrifuge tube (1.5 ml). The extracted protein (20–30 μl) was transferred into another centrifuge tube for later use. The 5× loading buffer of 1/4 volume was added to the remaining protein samples. The mixture was boiled for 5 min, followed by ice bath for 5 min immediately after. After the samples had been distributed to each group, they were kept under −20°C for later use. Following sodium dodecyl sulfate polyacrylamide gel electrophoresis (SDS-PAGE), the samples were transferred onto the polyvinylidene difluoride (PVDF) membrane and the membrane was blocked with tris-buffer saline Tween + 20 (TBST) containing 5% skimmed milk and was kept overnight at 4°C. The samples were then added with primary antibodies, including p53 (ab26, 1:1000, mouse antibody), p-53 (ab1431, 1:1000, rabbit antibody), p21 (ab109199, 1:1000, rabbit antibody), SUMO2/3 (ab109005, 1:3000, rabbit antibody), GADD45α (ab180768, 1:500, rabbit antibody), MDM2 (ab38618, 1:1000, rabbit antibody), CDK2 (ab32147, 1:2000, rabbit antibody), CDK4 (ab199728, 1:2000, rabbit antibody), MMP-2 (ab37150, 1:1000, rabbit antibody), CyclinB1 (ab2096, 1:500, rabbit antibody), HIF-1α (ab113642, 1:2000, mouse antibody), and GAPDH (ab8245, 1:1000, mouse antibody) purchased from Abcam Inc., (Cambridge, U.K.). The membrane was washed three times with TBST, 5 min each time. Then, in accordance with the different primary antibodies, goat anti-rabbit secondary antibody (ab6721, 1:2000 dilution, goat antibody) or goat anti-mouse secondary antibody (ab6785, 1:10000 dilution, goat antibody), purchased from Abcam Inc., (Cambridge, U.K.) was added and incubated at 37°C for 1 h. The membrane was then washed three times with TBST, 5 min each time, followed by the addition of 3-amino-9-ethylcarbozole (GK342011) for coloration. For gray value analysis, ImageJ was used according to the following equation: protein expression = target protein gray value/GAPDH internal gray value.

### 3-(4,5-dimethylthiazol-2-yl)2,5-diphenyl tetrazolium bromide (MTT) assay

The 35th generation NPCs in the sham, model, NC, and shRNA groups were seeded into a 96-well plate with 2 × 10^3^ cells per well and 24 wells per group. The cells were cultured in a cell incubator with saturated humidity and with 5% CO_2_ at 37°C. MTT assay was performed on the first, third, fifth, and seventh day of culture. MTT solution (20 μl, 5 mg/ml) was added into each well, and the cells were incubated at 37°C for 4 h. After removal of the supernatant, dimethyl sulfoxide (DMSO) (150 μl) was added into each well, followed by oscillation for 10 min. The growth curve was drawn according to the optical density (OD) value of each well at 450 nm.

### Flow cytometry

Flow cytometry was used in order to measure the cell cycle of the 35th generation NPCs in the sham, model, NC, and shRNA groups. After being washed with PBS, the cells were fixed in 70% ethanol and precooled at 4°C for at least 1 h. Cells were centrifuged at 1500 rev/min for 5 min for the removal of the fixative solution. The cell precipitate was washed once with PBS. Propidium iodide (PI) solution was added according to the instructions of DNA ploidy test kit (Sigma-Aldrich Chemical Company, St Louis MO, U.S.A.). The BD FACSVerse™ flow cytometry (Becton, Dickinson and Company, Franklin Lakes, NJ, U.S.A.) was used to detect cell cycle after 15 min, avoiding light. The DNA content per cell cycle was measured at 488 nm, with at least 10,000 cells counted each time.

The apoptosis of the 35th generation apoptotic NPCs in the sham, model, NC, and shRNA groups were examined. After the digestion of the cells in each group with trypsin without ethylenediaminetetraacetic acid (EDTA), centrifugation at 2000 rev/min for 5 min and washing twice with precooled PBS, the cells were collected and diluted with dye buffer to adjust cell density to 1 × 10^6^ cells/ml. The cells (100 μl) were then mixed with Annexin V-adenomatous polyposis coli (APC) (5 μl, Nanjing Kaiji, Nanjing, China) in an EP tube, followed by incubation for 15 min devoid of light. Subsequently, cells were tested by flow cytometry. The *E*_x_/*E*_m_ = 633/660 nm ratio was used to detect Annexin V-APC red fluorescence and the cell apoptosis was recorded.

### Senescence-associated β-galactosidase (SA-β-Gal) staining

The cell senescence of the 35th generation NPCs was detected in the sham, model, NC and shRNA groups. The cells in each group were seeded in a 24-well plate at a density of 4 × 10^4^ cells/well (6 wells per group). When the cells grew to 70% at the bottom of the bottle, they were washed with PBS. SA-β-gal staining solution was added to the cells according to the instructions of SA-β-gal staining kit (Beyotime Biotechnology Co., Shanghai, China). Cells were fixed at room temperature for 15 min. Following the removal of the fixed solution, the cells were washed three times with PBS, 3 min each time. SA-β-gal stained working solution was added and incubated at 37°C overnight, after which the cell was sealed with plastic wrap. Cell senescence was observed by an optical microscope.

### Statistical analysis

SPSS 22.0 statistical software (IBM Corp Armonk, NY, U.S.A.) was used for analysis. The measurement data were expressed as mean ± standard deviation (SD). Comparison of measurement data with normality and homoscedasticity between the two groups was analyzed using student’s *t*-test, while comparison of measurement data with normality and homoscedasticity among multiple groups was analyzed through a one-way factor analysis of variance (ANOVA). Comparison of measurement data without normality and homoscedasticity between two groups was analyzed using a rank-sum test. All experiments were repeated three times. With 0.05 regarded as the inspection level, a value of *P*<0.05 was considered to be statistically significant.

## Results

### Verification of IDD rats

The pathological changes in the intervertebral disc NPCs of rats in the sham and IDD groups were observed through HE stains. The results from the observations made under an optical microscope in the sham group revealed an intact intervertebral disc nucleus, thin fibrous plate, and proliferative chondrocytes. On the other hand, the NPCs of rats in the IDD group presented with proliferated intervertebral disc chondrocytes, disorderly arranged cartilage taking the place for fibrous plate, trabecular bone formation, blurred nucleus pulposus, and degenerated intervertebral disc.

In the sham group, the normal cartilage-like cells were observed by an electron microscopy with normal organelle, and the cell membrane was intact and smooth with no calcination of fine particles with high electron density. Collagen fiber was arranged regularly and fitly without mass structure and cross-linking. Cells in the IDD group were irregularly arranged, degenerated, or died, in which abundant heterochromatin in the nucleus, reduced organelles, and calcination of fine particles with high electron density was observed. The collagen fiber presented with a myelin-like or wool-like, and stacked into pieces or fingerprint structure, which was degenerated and intertwined. The edge was rough and blurred with disappeared stripes, and a blurry internal structure (Figure 1).

**Figure 1:** The HE staining reflects pathological changes in NPCs of IDD rats under the optical microscope and electron microscope Under the optical microscope, the chondrocytes were irregularly arranged, and the NPCs were disrupted in the rats with IDD. In addition, under the electron microscope, degenerated NPCs, some microcalcifications with high electron density, and sheath or wool-like collagen fibrils were observed in the rats with IDD; HE, hematoxylin and eosin; IDD, intervertebral disc degeneration; NPC, nucleus pulposus cell.

### Higher positive expressions of SUMO2/3 proteins in the NP of IDD rats

The results revealed that IDD rats showed higher positive expression of SUMO2/3 protein.

Immunohistochemistry was adopted to detect the positive expression of SUMO2/3 protein in mice in the sham and IDD groups. The brown particles of SUMO2/3 protein were found in the nucleus pulposus tissues of rats in both the model and sham groups, suggesting that SUMO2/3 protein expressions were positive. The positive expression of SUMO2/3 protein in the IDD group was also found to be higher than that in the sham group (Figure 2).

**Figure 2:** SUMO2/3 protein expressed in NPCs between the sham and IDD group, determined by immunohistochemistry (**A**) SUMO2/3-positive cells were brown-stained, which were pointed by black arrows (×400). (**B**) Quantitative analysis of SUMO2/3-positive cells; *P<0.05, compared with the sham group; IDD, intervertebral disc degeneration; NPC, nucleus pulposus cell; SUMO, small ubiquitin-related modifier.

### Reduced type II collagen-positive NPCs in IDD rats

The phenotypic molecule expression of NPCs in rats in the sham and IDD groups was detected. The expression of type II collagen in the 2nd generation NPCs in the sham and IDD groups was found to be positive. The cytoplasm could be stained to a brownish yellow appearance, while the nucleus wasn’t able to do so. It was also observed that the expression of type II collagen in the 2nd generation NPCs in sham group was higher than that in IDD group (Figure 3). Based on these results, it was known that IDD rats showed poor phenotypic molecules expressions of NPCs.

**Figure 3:** Expressions of type II collagen in NPCs in the sham and IDD groups, determined by optical microscope Notes: IDD, intervertebral disc degeneration; NPC, nucleus pulposus cell.

### Morphology of NPCs in IDD rats

The changes in the growth morphology of NPCs in rats in the sham and IDD groups were observed. The primary NPCs (Figure 4A) of the sham group began to adhere to the wall 2–3 days after inoculation with round shape. The passage cells (Figure 4C) gradually extended into polygonal or short spindle shape. The appearance presented to be paving stone shape and fully covering the bottom of the bottle 7–9 days after inoculation. The primary NPCs from rats in the IDD group (Figure 4B) grew slowly with low adherence rate. Following inoculation for 5–6 days, cells were adhered to the wall and reached the confluence state 12–14 days after inoculation. It was observed that the passage cells (Figure 4D) were homogeneous, typical of polygonal or short spindle. The nucleus presented to have a larger oval shape with clear outline. There were multiple nucleoli in cells and the cell body was flatter and larger. The nuclear grew in size, while the refractive power of cytoplasm weakened. These findings revealed that IDD rats displayed obvious changes in their growth morphology in NPCs.

**Figure 4:** Obvious changes of growth morphology were observed in IDD rats under the transmission electron microscope Notes: Primary sham group (×40). Primary IDD group (×40). Passage sham group (×100). Passage IDD group (×100); NPC, nucleus pulposus cells; IDD, intervertebral disc degeneration.

### Lentiviral-mediated silencing SUMO2

The lentivirus vectors were constructed in order for the detection of green fluorescence in NPCs in each group. In NPCs in the PLL-SUMO2-shRNA1, PLL-SUMO2-shRNA2 and PLL-SUMO2-shRNA3 groups, a stronger green fluorescence observed under a fluorescence microscope. There was no significant difference among three groups, while NPCs in the PBS group showed no green fluorescence (Figure 5). The results indicated higher expression of green fluorescent protein in the three PLL-SUMO2-shRNA groups.

**Figure 5:** GFP gene report shows higher expression of green fluorescent protein in the three PLL-SUMO2-shRNA groups by fluorescence microscopy Notes: GFP, green-fluorescent protein; SUMO, small ubiquitin-related modifier.

### SUMO2 modulates the p53 signaling pathway

The qRT-PCR and Western blotting were adopted to determine mRNA and protein levels of SUMO2, p53, p21, MDM2, GADD45α, MMP-2, HIF-1α, CDK2/4, and CyclinB1 and p53 phosphorylation level of NPCs of rats in each group. Compared with the sham group, the mRNA level of SUMO2 of NPCs in the remaining groups was up-regulated, and the mRNA level of SUMO2 of NPCs in the model and NC groups was significantly higher than that in the sham group (*P*<0.05). The SUMO2 mRNA level in the shRNA1, shRNA2, and shRNA3 groups was significantly lower than that of the IDD group (*P*<0.05), and the lowest SUMO2 mRNA level among the shRNA1, shRNA2, and shRNA 3 groups was the shRNA3 group, which was selected as the shRNA group with the highest silencing efficiency (*P*<0.05). Compared with sham group, the mRNA and protein levels of SUMO2, MMP-2, HIF-1α, and p53 signaling pathway-related genes (p53, p21, MDM2, and GADD45α) of NPCs in other groups were increased, while the mRNA and protein levels of p53 signaling pathway-related genes CDK2/4 and CyclinB1 decreased. The mRNA and protein levels of SUMO2, p53, p21, MDM2, GADD45α, MMP-2, and HIF-1α, and the p53 phosphorylation level of NPCs in the shRNA group were significantly lower than those in the IDD group (*P*<0.05), but the mRNA and protein levels of CDK2/4 and CyclinB1 were significantly higher than that in the IDD group (*P*<0.05). There was no significant difference observed between the model and NC group (*P*>0.05) (Figure 6). All of the aforementioned findings revealed that SUMO2 gene silencing reduces the levels of SUMO2, p53, p21, MDM2, GADD45α, MMP-2, and HIF-1α expressions and p53 phosphorylation level but elevates the levels of CDK2/4 and CyclinB1 expressions.

**Figure 6:** The results from RT-qPCR and Western blotting demonstrate that SUMO2 gene silencing decreases the levels of SUMO2, p53, p21, MDM2, GADD45α, MMP-2, and HIF-1α expressions and p53 phosphorylation level but increases the levels of CDK2/4 and CyclinB1 expression Notes: (**A**) mRNA level of SUMO2 in the six groups. (**B**) mRNA levels of SUMO2/3, p53, p21, MDM2, CDK2/4, CyclinB1, MMP-2, and HIF-1α in the sham, model, NC and shRNA group. (**C**) Gray values of SUMO2/3, p53, p21, GADD45α, MDM2, CDK2/4, CyclinB1, MMP-2, and HIF-1α. (**D**) Protein levels of SUMO2/3, p53, p21, GADD45α, MDM2, CDK2/4, CyclinB1, MMP-2, and HIF-1α in the sham, model, NC and shRNA groups; *P<0.05, compared with the sham group; ^#^*P*<0.05, compared with the model and NC groups; CDK2/4, cyclin-dependent kinase 2/4; GADD45α, growth arrest and DNA damage inducible 45α; HIF-1α, hypoxia-inducible factor-1α; MDM2, mouse double minute 2; MMP-2, matrix metalloproteinase-2; NC, negative control; RT-qPCR, reverse transcription quantitative polymerase chain reaction; SUMO2/3, small ubiquitin-related modifier 2/3.

### Silencing SUMO2 enhances proliferation of NPCs

MTT assay was performed to detect viability of NPCs in each group. As shown in Figure 7, there was no significant difference in proliferation of the 35th generation cells in each group on the first, third, and fifth day. However, compared with the sham group, with increasing incubation time, the proliferation rate of NPCs in other groups decreased with different degrees with decreased proliferation, prolonged cell latency, and slacken logarithmic growth phase. The proliferation of NPCs in the model, NC, and shRNA groups were significantly lower than that of the sham group on the seventh day (*P*<0.05), and the proliferation of NPCs in the shRNA group was significantly higher than that in the IDD group (*P*<0.05). There was no significant difference between the model and NC groups (*P*>0.05). These results showed that SUMO2 gene silencing promotes the proliferation of NPCs.

**Figure 7:** The MTT assay shows that SUMO2 gene silencing enhances proliferation of NPCs Notes: *P<0.05, compared with the sham group; ^#^*P*<0.05, compared with the model and NC groups; MTT, 3-(4,5-dimethylthiazol-2-yl)2,5-diphenyl tetrazolium bromide; NC, negative control; OD, optical density.

### Silencing SUMO2 promotes cell cycle entry of NPCs

Flow cytometry of PI staining was employed to detect cell cycle entry of NPCs. As shown in Figure 8, compared with the sham group, the proportion of NPC in the G1 and G2 phase of the 35th generation cells in the other groups increased, while the proportion of NPCs in the S phase decreased. The proportion of NPCs in the G1 phase of model and the NC group was significantly higher than that in the sham group (*P*<0.05), and the proportion of NPCs in the S phase of model and NC group was significantly lower than that in the sham group (*P*<0.05). The proportion of NPCs in the G1 phase of shRNA group was significantly lower than that of IDD group (*P*<0.05), while the proportion of NPCs in the S phase of shRNA group was significantly higher than that of the IDD group (*P*<0.05). Compared with the sham group, the proportion of NPCs in the G2 phase of the other groups was higher, but the change was not statistically significant. There was no significant difference between model and NC groups (*P*>0.05). These findings indicated that SUMO2 gene silencing promotes cell cycle entry in NPCs.

**Figure 8:** Flow cytometry analysis of PI staining shows that SUMO2 gene silencing promotes cell cycle entry of NPCs Notes: (**A**) Cell cycle entry of NPCs in the sham, model, NC, and shRNA groups. (**B**) Percentage chart of cell cycle of NPCs in the sham, model, NC, and shRNA groups; *P<0.05, compared with the sham group; ^#^*P*<0.05, compared with the model and NC groups; NC, negative control; NPC, nucleus pulposus cell; PI, propidium iodide.

### Silencing SUMO2 inhibits apoptosis of NPCs

Apoptosis of NPCs was detected by flow cytometry of Annexin V-APC staining. As shown in Figure 9, compared with the sham group, the apoptotic rate of the 35th generation cells in the remaining groups were higher (*P*<0.05). The apoptotic rate in the model and NC groups was obviously higher than in the sham group (*P*<0.05). The apoptotic rate in the shRNA group was obviously lower than that in IDD group (*P*<0.05). There was no significant difference between the model and NC groups (*P*>0.05). These findings revealed that SUMO2 gene silencing inhibits apoptosis of NPCs.

**Figure 9:** Flow cytometry analysis of Annexin V-APC staining shows that SUMO2 gene silencing inhibits apoptosis Notes: (**A**) Apoptosis of NPCs in the sham, model, NC, and shRNA groups. (**B**) Apoptotic rate of NPCs in the sham, model, NC, and shRNA groups; *P<0.05, compared with the sham group; ^#^*P*<0.05, compared with the model and NC groups; Annexin V-APC, Annexin V- adenomatous polyposis coli; NC, negative control; NPC, nucleus pulposus cell.

### Silencing SUMO2 suppresses senescence of NPCs

The SA-β-gal staining was adopted to detect senescence of NPCs. As shown in Figure 10, the positive rate of SA-β-gal staining of the 35th generation cells found to be higher in the remaining groups in comparison with the sham group. The nucleus in the sham group did not appear to be stained following SA-β-gal staining. Cytoplasm in the sham group had a dark blue appearance, and was found without vacuole. However, some of the nucleus pulposus cytoplasm appeared to be dark blue in color, and there were obvious vacuoles in the model, NC, and shRNA groups. The positive rate of cell senescence in the model and NC groups was significantly higher than that in the sham group (*P*<0.05). The positive rate of cell senescence in the shRNA group was significantly lower than that in the IDD group (*P*<0.05). There was no significant difference between the model and NC groups (*P*>0.05). These results showed that SUMO2 gene silencing suppresses senescence of NPCs.

**Figure 10:** The SA-β-gal staining revealed that SUMO2 gene silencing suppresses senescence of NPCs Notes: (**A**) SA-β-gal staining observation of NPCs in the sham, model, NC, and shRNA groups (×400). (**B**) SA-β-gal staining positive rate of NPCs in the sham, model, NC, and shRNA groups; *P<0.05, compared with the sham group; #*P*<0.05, compared with the model and NC groups; NC, negative control; NPC, nucleus pulposus cell; SA-β-gal, senescence-associated β-galactosidase.

## Discussion

IDD is a complex phenomenon implicated by lower back pain and is a prerequisite to disk herniation, which begins early in life and is caused by various intrinsic and extrinsic factors as well as normal aging [15,16]. SUMOs have been considered to be versatile regulators of many biological functions [17]. Moreover, it has previously been reported that p53 pathway plays a significant role in the senescence of CEP cells, which is one of the components of IDD [11]. Therefore, our study was conducted aiming to investigate the ability of SUMO2 gene silencing in the stimulation of the proliferation, apoptosis, and senescence of NPCs through the p53 signaling pathway mediation in IDD rats.

Our findings revealed that the positive SUMO2/3 protein expression in the IDD group was higher in comparison with the sham group, while the expression of type II collagen showed the opposite results. The combination of matrix in IDD is a result of the change of production of collagen including type II and type I in the nucleus pulposus and inner annulus fibrosus [18]. It is known that IDD is caused by the enzymatic breakdown of extracellular matrix and possibly local inflammation [16]. SUMO1-3 are proteins associated with ubiquitin which are involved in the process of post-translational modification of lysine residues of target proteins including SUMO-specific activating, conjugating, and ligating enzymes [19]. A study by Deng et al. [20] has demonstrated that Ubc9, a specific SUMO-conjugating enzyme, is also highly activated in tumor cells, which was found to be consistent with our study. In addition, the findings also showed that the matrix in IDD rats affects type II collagen expression in the IDD group and it was lower in comparison with the sham group.

In addition, the mRNA and protein levels of SUMO2, p53, p21, MDM2, GADD45α, and the phosphorylation level of p53 in the shRNA groups were obviously lower than those in the IDD group, while the mRNA and protein levels of CDK2/4 and CyclinB1 showed a reverse trend. The modification of SUMO-2 was proved to regulate p53 in human embryonic kidney 293 cells [21]. It is known that p53, p21, MDM2, and GADD45α are closely related to the p53 signaling pathway [22–24]. In addition, according to Stindt et al., p53 is activated by post-translational modification, including modification by SUMO [25]. Thus, it is reasonable to draw the conclusion that the p53 signaling pathway-related expressions were regulated by SUMO-2/3, and high expression level of SUMO-2/3 in IDD rats promoted the mRNA and protein expressions of p53. In addition, it is known that MDM2 targeted p53 to the nucleolus by the formation of the MDM2/p53 complex and promoted p53 sumoylation [26]. These results were all consistent with our conclusion.

The proliferation rate of NPCs in the shRNA group was higher than that in the IDD group, while the senescence and apoptotic rates were significantly lower, suggesting that while the SUMO gene silencing promoted cell proliferation, it inhibited cell senescence and apoptosis. The apoptosis and senescence of NPCs are the fundamental pathological findings in IDD [27]. Cell senescence is also regarded as a relevant element in human disc degeneration [28]. Therefore, the apoptosis rate was elevated in the IDD group. Also p53 modified by SUMO-2/3 might be a stress response signal, and it may promote the expression of target genes, and thereby results in cellular responses like senescence [21], which could explain the low senescence rate in the shRNA groups. Moreover, it has been reported that SUMO-1 can enhance the HepG2 cell apoptosis induced by wild-type p53 as it binds to p53 protein [29].

According to the results of our study, SUMO2 could serve as a potential therapeutic target for the following reasons. First, down-regulation of SUMO2 could enhance proliferation, and suppress apoptosis and senescence of NPCs. Second, the inhibition of p53 signaling pathway is responsible for the beneficial effects of SUMO2 inhibition on NPCs. To our knowledge, our findings for the first time revealed the involvement of SUMO molecules in IDD pathogenesis. However, the underlying mechanisms on how SUMO2 gene silencing promoted proliferation and inhibited the apoptosis and postponed senescence of NPCs through the p53 signaling pathway, as well as the potential mechanism in cell apoptosis and senescence of NPCs in IDD rats were not thoroughly identified. Therefore, more studies need to be conducted for further investigations.

## Abbreviations

AF: anulus fibrosus
CDK2/4: cyclin-dependent kinase 2/4
CEP: cartilage end plate
DAB: diaminobenzidine
GADD45α: growth arrest and DNA-damage-inducible protein 45 α
HIF-1α: hypoxia-inducible factor-1α
IDD: intervertebral disc degeneration
MDM2: murine double minute-2
MMP-2: matrix metalloproteinase-2
NPC: nucleus pulposus cell
PI: propidium iodide
SUMO: small ubiquitin-related modifier
